The article "Exploring the Effect of Enbrel Softgels on PWI Indicators in VCIND Patients" was retracted in 2023. Reasons: signs of a paper mill; suspected computer-generated content; unreliable results or conclusions; concerns about the data.

# Exploring the Effect of Enbrel Softgels on PWI Indicators in VCIND Patients

**DOI:** 10.1155/2022/9681235

**Published:** 2022-04-06

**Authors:** Lei Cui, Pan Li, Jingchen Zhang, Xiaofang Li

**Affiliations:** ^1^Department of Neurology, Affiliated Hospital of Hebei University, Baoding, Hebei 071000, China; ^2^Department of Neurology, Baoding No. 1 Central Hospital, Baoding, Hebei 071000, China

## Abstract

**Objective:**

To investigate the effect of Enbrel softgels on the head nuclear magnetic (PWI) indices in patients with vascular cognitive impairment-no dementia (vascular cognitive impairment-no dementia, VCIND).

**Methods:**

Patients with confirmed VCIND hospitalized in the Department of Neurology of the Affiliated Hospital of Hebei University from April 2017 to April 2019 were included in the study, and they were divided into experimental and control groups (30 patients in each group) according to the difference of interventions. The PWI examination and neuropsychological assessment were performed at the beginning of the experiment, 12 w after treatment, and 48 w after treatment in the two groups. Score differences between the two groups and the preliminary demonstration of the clinical value of the MMSE and ADAS-Cog in the diagnosis of VCIND.

**Results:**

(1) The difference in PWI positivity rate between the two groups at the beginning of the experiment was not statistically significant (*P* > 0.05); the PWI positivity rate in the experimental group at 12 W was significantly lower than that in the control group (*P* < 0.05); the difference in PWI positivity rate between the two groups at 48 W was not statistically significant (*P* < 0.05); (2) the MMSE scores of patients in the experimental group at 12 W and 48 W were higher than those in the control group, and the ADAS-Cog scores were lower than those in the control group (*P* < 0.05). (3) The diagnostic AUCs of MMSE and ADAS-Cog for VCIND were 0.7960 (95% CI = 0.6411–0.9508, *P*=0.0037) and 0.9291 (95% CI = 0.8390), respectively (95% CI = 0.8390–1.000, *P* < 0.0001).

**Conclusion:**

The addition of Enbrel softgels to concomitant therapy in VCIND patients can lead to changes in their PWI imaging indicators, which in turn can have a significant impact on their neuropsychological indicators, and quantitative analysis scales such as the MMSE and ADAS-Cog can be considered for the diagnostic treatment of VCIND.

## 1. Introduction 

Vascular cognitive impairment-no dementia (VCIND) is a cognitive dysfunction due to cerebrovascular disease, generally ischaemic cerebrovascular lesions [1]. Patients can present with dysfunction in multiple or single cognitive domains such as visuospatial and executive abilities, memory, attention, language, abstraction, calculation, and orientation [2, 3]. These cognitive dysfunctions are often partially impaired and do not meet the diagnostic criteria for dementia, and the patient's ability to perform daily life is generally unaffected [4]. With the development of an ageing population and longer life expectancy in our society, the incidence of cerebrovascular disease is increasing, and the corresponding incidence of vascular cognitive dysfunction is also on the rise [5].

The article "Exploring the Effect of Enbrel Softgels on PWI Indicators in VCIND Patients" was retracted in 2023. Reasons: signs of a paper mill; suspected computer-generated content; unreliable results or conclusions; concerns about the data.

There is no effective drug to cure vascular cognitive dysfunction, but the symptoms of cognitive impairment can be further improved by controlling the risk factors of cerebrovascular disease and carrying out postischemic neuroprotective treatment to improve the quality of survival and delay the progression of the disease [6, 7]. Enbrel soft capsule is a new class I drug developed independently in China for the treatment of ischaemic stroke, and has been widely used in the acute clinical treatment of ischaemic cerebrovascular disease in recent years [8]. PWI is the most important clinical test for the diagnosis of intracranial lesions, which can calculate cerebral blood volume (rCBV), local cerebral blood flow (rCBF), and mean time to passage (MTT). It shows the blood flow in the capillary network, which in turn provides the functional status of oxygen and nutrients in the surrounding tissues and is used in the diagnosis and assessment of disease [9, 10]. In this paper, we propose to investigate the changes in PWI indicators after the application of Enbrel softgels to patients with VCIND by setting up a control group in order to provide a new reference for the clinical treatment and diagnostic assessment of these patients.

## 2. Materials and Methods

### 2.1. General Information

Patients with confirmed VCIND hospitalized in the Department of Neurology of the Affiliated Hospital of Hebei University from April 2017 to April 2019 were included in the study, and they were distinguished into experimental and control groups (30 patients in each group) according to the differences in interventions.

#### 2.1.1. Inclusion Criteria

The inclusion criteria were as follows: (1) neuropsychological assessment of patients with cognitive impairment but not at the level of dementia; (2) MMSE ≥24 in the junior high school and above group and ≥20 in the primary school group (MMSE ≤28); (3) MRI of the head showing subcortical ischaemic vascular disease; and (4) age 60–75 years.

#### 2.1.2. Exclusion Criteria

The exclusion criteria were as follows: (1) those with severe psychiatric or neurological disorders who cannot cooperate with the neuropsychological assessment examination; (2) those with other disorders affecting cognitive function or cognitive impairment due to drug dependence; (3) those with severe psychiatric disorders; (4) those with new cerebral infarction within 3 months prior to enrolment; (5) those with severe gastrointestinal, circulatory, urinary, and immune system disorders; (6) those who are allergic to the investigational drug; and (7) those who are unable to complete the head MRI.

The article "Exploring the Effect of Enbrel Softgels on PWI Indicators in VCIND Patients" was retracted in 2023. Reasons: signs of a paper mill; suspected computer-generated content; unreliable results or conclusions; concerns about the data.

### 2.2. Research Method

After admission, patients in both groups received conventional interventions, such as the application of drugs to improve cerebral blood flow, the start of hyperbaric oxygen chamber therapy, and the application of neurotrophic factors. Meanwhile, the control group was given nimodipine (manufacturer: Yabao Pharmaceutical Group Co., Ltd., specification 20 mg/tablet, and approval number: State Drug Quantifier H14022821) 30 mg/time, 3 times daily, for 90 days. The experimental group was supplemented with Enbep Soft Capsules (trade name: Butylphthalein Soft Capsules, manufacturer: Shiyang Pharmaceutical Group, Enbep Pharmaceutical Co., Ltd., specification 0.1 g/capsule, and approval number: Guo medicine quantity H20050299) 200 mg/dose, 3 times daily for 90 days.

### 2.3. Observational Indicators and Rubrics

#### 2.3.1. Neuropsychological Scores

Neuropsychological scores were administered before the start of the trial, at 12 weeks of treatment, and at 48 weeks after treatment, using the MMSE and ADAS-cog scales, respectively. The staff conducting the assessments were trained and tested before the start of the trial to ensure the objectivity of the results. The scales were assessed in a dedicated neurology laboratory in a quiet and relaxed environment. The MMSE scale [11] is the most widely used cognitive screening scale both nationally and internationally, covering orientation, memory, attention, numeracy, language skills, and visuospatial abilities. The scale covers a wide range of topics but is relatively simple to administer and easy for the assessing practitioner to master. The total score ranges from 0 to 30, with higher scores indicating better cognitive functioning. However, the MMSE scale has limitations in differentiating normal elderly people from those with mild cognitive impairment. Therefore, this experiment also assessed patients on the ADAS-cog scale [12], which consists of 12 items covering memory, orientation, language, use, and attention and can assess the severity of cognitive symptoms and treatment changes in patients. In this trial, five subtests reflecting attention/executive function, including digit breadth (backwards recall), digit scratching, symbolic digit conversion, verbal fluency, and maze test, were added to it to further assess vascular cognitive impairment.

The article "Exploring the Effect of Enbrel Softgels on PWI Indicators in VCIND Patients" was retracted in 2023. Reasons: signs of a paper mill; suspected computer-generated content; unreliable results or conclusions; concerns about the data.

#### 2.3.2. Head MRI (PWI)

PWI (PWI parameters: SE-EPI sequence, TR 1500 ms, TE 16 ms, layer thickness set to 4 mm, spacing set to 0 mm, contrast agent injected via elbow vein using a high-pressure syringe, 0.15 ml/kg injected according to body weight, and flow rate set to 4 ml/s) was used to investigate brain perfusion in the two groups of patients at the beginning of the experiment, 12 W of the experiment, and at 48 W of the experiment. The patients with reduced perfusion in the PWI study area were defined as positive, and the difference in the rate of positive PWI between the two groups at different observation times was recorded.

### 2.4. Statistical Methods

The SPSS22.0 statistical software was chosen to analyse the data collected in the study, in which the measures were expressed as mean ± standard deviation, and the tests of normal distribution and chi-square were carried out. The difference between groups was tested using the chi-square test and the diagnostic value was analyzed using the ROC curve, with *P* < 0.05 being taken as a statistically significant difference. Graphpad prism 8.3 was used for this study [13].

## 3. Results

### 3.1. Comparison of the Differences in Baseline Clinical Information between the Two Groups

The gender, age, and previous disease history of the two groups were included in the study, and a comparison of the differences between the groups was implemented. The results showed that the differences between the groups in terms of the above baseline clinical information were not statistically significant (*P* > 0.05), suggesting that the two groups were comparable (Table 1).

### 3.2. Analysis of the Changes in PWI Indicators before and after the Intervention in the Two Groups

The PWI test was carried out at the beginning of the experiment at w 12 and w 48 for the two groups of patients, respectively, and the positive rate of PWI in the group at different observation times was recorded and compared between the groups (0.05). At 12 w after treatment, there was 1 positive PWI case in the experimental group, with a positive rate of 3.33%, and 7 positive PWI cases in the control group, with a positive rate of 23.33%, with a significant difference between the two groups (*P* < 0.05). At 48 w after treatment, there was 1 positive PWI case in the experimental group, with a positive rate of 3.33%, and 5 positive PWI cases in the control group, with a positive rate of 16.67%, with no significant difference between the two groups (*P* > 0.05) (Table 2 and Figure 1) and Figure 2.

### 3.3. Comparison of Neuropsychological Scores between the Two Groups of Patients before and after the Intervention

The neuropsychological functioning of the two groups was assessed using the MMSE and ADAS-Cog scores at the beginning of the experiment, at experiment 12 W and at experiment 48 W, respectively, and the differences between the groups were compared. The results showed that the difference between the two groups of patients' MMSE scores at the beginning of the experiment was not statistically significant (*P* > 0.05), and the MMSE scores of the patients in the experimental group were significantly higher than those of the control group at both the 12th W and 48th W of the experiment, and the difference between the groups was statistically significant (*P* < 0.05). The MMSE scores were higher in the experimental group than at the beginning of the experiment at both the 12th W and 48th W of the experiment (*P* < 0.05), while the difference was not statistically significant in the control group before and after the comparison (*P* > 0.05). The difference in ADAS-cog scores between the two groups at the beginning of the experiment was not statistically significant (*P* > 0.05), while the ADAS-cog scores of patients in the experimental group were significantly lower than those in the control group at both the 12th W and 48th W of the experiment, and the difference between the groups was statistically significant (*P* < 0.05). The ADAS-cog scores were lower in the experimental group than at the beginning of the experiment at both the 12th W and 48th W of the experiment in the within-group comparison (*P* < 0.05), while the difference was not statistically significant in the control group before and after the comparison (*P* > 0.05) (Table 3 and Figure 3).

The article "Exploring the Effect of Enbrel Softgels on PWI Indicators in VCIND Patients" was retracted in 2023. Reasons: signs of a paper mill; suspected computer-generated content; unreliable results or conclusions; concerns about the data.

### 3.4. Analysis of the Diagnostic Value of MMSE and ADAS-Cog Scores for VCIND

The diagnostic ROC curves for the MMSE and ADAS-cog scores for VCIND were plotted separately, and their AUCs were calculated, showing AUCs of 0.7960 (95% CI = 0.6411–0.9508, *P*=0.0037) and 0.9291 (95% CI = 0.8390–1.000, *P* < 0.0001) for the above scales, respectively (Figure 4).

## 4. Discussion

In recent years, the incidence of dementia has increased year by year as the population ages [14]. Currently, approximately about 30 million people worldwide suffer from dementia, and it is expected that this number will increase to 42 million by 2021 [15]. Vascular injury is the second most common cause of dementia, with subcortical ischaemic cerebrovascular disease, typically caused by lacunar infarction or white matter injury, being the most common cause of vascular cognitive impairment [16]. Vascular nondementia cognitive impairment (VCIND) refers to early or mild cognitive impairment due to vascular injury, a state of cognitive impairment between normal individuals and dementia, and is generally considered to be the early stage of vascular cognitive impairment, with a variety of risk factors that are highly intervenable. The incidence of dementia is also significantly reduced if appropriate interventions are provided [17, 18]. Studies have shown that approximately 40% of patients with VCIND progress to vascular dementia within 2 years, and those who have progressed to vascular dementia experience irreversible deterioration [19], so appropriate intervention and treatment of patients with VCIND can help improve the prognosis and quality of life of older people with vascular injury.

The article "Exploring the Effect of Enbrel Softgels on PWI Indicators in VCIND Patients" was retracted in 2023. Reasons: signs of a paper mill; suspected computer-generated content; unreliable results or conclusions; concerns about the data.

Enbep softgel is a butanol-based soft gel capsule commonly used in the treatment of mild to moderate acute ischaemic stroke. It has been shown to have a variety of pharmacological effects and to be a comprehensive treatment for the symptoms of neurological deficits caused by ischaemic stroke, with positive implications for improving the patient's ability to live [20]. In this study, the effect of Enbrel soft gelatin capsules on the PWI index of VCIND patients was analyzed by establishing a control group. The results showed that compared to the control group, the experimental group with Enbrel soft gelatin capsules showed a significant decrease in the PWI positivity rate at 12 weeks of treatment compared to the beginning of the experiment, and the PWI positivity rate at 12 weeks of treatment was significantly lower than that of the control group, which This suggests that the intervention effect of Enbrel softgels was significant, which is consistent with the findings of other scholars. A study conducted on 58 patients with chronic cerebral insufficiency showed that Enbep Soft Capsules had a good clinical intervention effect on chronic cerebral insufficiency, and patients treated with the drug showed significant improvement in transcranial Doppler ultrasound indices [21]. The authors of this paper analyzed that butyl-phenol is a chemical component that can protect brain tissue in multiple ways. This substance can use the increase of nitric oxide and prostaglandin in the cerebrovascular endothelium to reduce intracellular calcium concentration, thus achieving the effect of inhibiting glutamate release and inhibiting oxygen free radical damage to brain cells, and also improving ischaemic and hypoxic symptoms by increasing microcirculation and blood flow in the ischaemic areas of brain tissue, with multiple mechanisms. It can also improve the symptoms of ischemia and hypoxia by increasing microcirculation and blood flow in the ischaemic area of brain tissue and improving the impaired functional state of brain tissue brought about by vascular injury through multiple mechanisms [22].

The article "Exploring the Effect of Enbrel Softgels on PWI Indicators in VCIND Patients" was retracted in 2023. Reasons: signs of a paper mill; suspected computer-generated content; unreliable results or conclusions; concerns about the data.

The paper further demonstrates the effect of Enbrel softgels on the neurobiological indicators of VCIND patients. The data show that the MMSE scores of the patients in the experimental group were higher than those of the control group, and the ADAS-cog scores were lower than those of the control group at both time points, 12 and 48 weeks after receiving the experiment, suggesting that the use of Enbrel softgels effectively improved the neurological function of VCIND patients and also improved the clinical manifestations of Alzheimer's disease. A randomized controlled study conducted on 178 acute stroke patients found that the application of Enbrel capsules reduced the incidence of poststroke dementia from 14.61% to 5.62% and improved the patients' cognitive function scores from (24.20 ± 4.43) to (25.30 ± 2.79) and behavioral ability scores from (52.40 ± 17.70) to (57.10 ± 13.30), a significant change [23]. Current animal experiments have demonstrated that butanol has a strong anti-cellular ischaemic-hypoxic effect, reduces the infarct area of local cerebral ischemia in rats, inhibits neuronal apoptosis, and inhibits thrombus formation, which the authors of this paper suggest is an important reason why Enbrel capsules can improve neurobiological scores in VCIND patients [24]. Finally, the paper also verified the value of MMSE and ADAS-cog scores in VCIND patients by plotting ROC curves, and the results suggested a better diagnostic value, which may provide a new reference for the clinical identification of VCIND patients.

In summary, the addition of Enbrel softgels to concomitant therapy in VCIND patients can lead to changes in their PWI imaging indicators, which in turn can have a significant impact on their neuropsychological indicators, and quantitative analysis scales such as the MMSE and ADAS-Cog can be considered for use in the diagnostic treatment of VCIND.

## Figures and Tables

**Figure 1:** Analysis of the changes in PWI indicators before and after the intervention in the two groups The difference in DWI positivity between the two groups at the beginning of the experiment was not statistically significant (*P* > 0.05), the DWI positivity rate in the experimental group was significantly lower than that in the control group at the 12th W of the experiment (*P* < 0.05), and the difference in DWI positivity between the two groups at the 48th week of the experiment was not statistically significant (*P* > 0.05).

**Figure 2:** Comparison of MMSE scores between the two groups before and after the intervention. The comparison showed that the difference between the two groups of patients' MMSE scores before the experiment was not statistically significant (*P* > 0.05), while the MMSE scores of the experimental group were higher than those of the control group at both the 12th W and 48th W of the experiment (*P* < 0.05) (a). Within the group, prepost variability was compared, with the experimental group (b) having higher MMSE scores at both the 12th W and 48th W than at the beginning of the experiment (*P* < 0.05), while the control group (c) did not have statistically significant differences in prepost comparisons (*P* > 0.05). # represents a statistically significant difference (Table 4).

The article "Exploring the Effect of Enbrel Softgels on PWI Indicators in VCIND Patients" was retracted in 2023. Reasons: signs of a paper mill; suspected computer-generated content; unreliable results or conclusions; concerns about the data.

**Figure 3:** Comparison of ADAS-cog scores between the two groups before and after the intervention. The comparison showed that the difference between the two groups in ADAS-cog scores before the experiment was not statistically significant (*P* > 0.05), and the ADAS-cog scores in the experimental group were lower than those in the control group at both the 12th W and 48th W of the experiment (*P* < 0.05) (a) Within-group, prepost variability was compared, with the experimental group (b) having lower ADAS-cog scores at both the 12th W and 48th W than at the beginning of the experiment (*P* < 0.05), while the control group (c) had no statistically significant differences in prepost comparisons (*P* > 0.05). # represents a statistically significant difference.

**Figure 4:** Analysis of the diagnostic value of MMSE and ADAS-cog scores for VCIND. The diagnostic AUC for VCIND was 0.7960 (95% CI = 0.6411–0.9508, *P*=0.0037) and 0.9291 (95% CI = 0.8390–1.000, *P* < 0.0001) for MMSE and ADAS-cog scores, respectively.

**Table 1:** Comparison of baseline information between the two groups of patients $\left(\bar{x}\pm s\right)/\left[n\left(\%\right)\right]$.

General clinical information		Experimental group (*n* = 30)	Control group (*n* = 30)	*t*/*χ*^2^	*P*
Gender	Male	18	17	0.069	0.793
	Female	12	13		

Average age (years)		69.57 ± 3.41	69.17 ± 3.01	0.482	0.632
Average weight (kg)		70.19 ± 2.39	69.98 ± 3.01	0.229	0.766
With or without medical insurance	Yes	27	28	0.218	0.64
	None	3	2		

High blood pressure	Yes	6	5	0.111	0.739
	None	24	25		

Diabetes	Yes	4	5	0.131	0.718
	None	26	25		

High blood cholesterol	Yes	7	8	0.089	0.766
	None	23	22		

Coronary heart disease	Yes	4	7	1.002	0.317
	None	26	23		

**Table 2:** Analysis of the changes in PWI indicators before and after the intervention in the two groups [*n*(%)].

Group	Number of examples	Start of the experiment	Experiment 12 w	Experiment 48 w
Experimental group	30	6(20.00)	1(3.33)	1(3.33)
Control group	30	7(23.33)	7(23.22)	5(16.67)
*χ* ^2^	—	0.098	5.192	2.963
*P*	—	0.754	0.023	0.085

The article "Exploring the Effect of Enbrel Softgels on PWI Indicators in VCIND Patients" was retracted in 2023. Reasons: signs of a paper mill; suspected computer-generated content; unreliable results or conclusions; concerns about the data.

**Table 3:** Comparison of MMSE scores between the two groups before and after the intervention ($\bar{x}\pm s$).

Group	Number of examples	Start of the experiment	Experiment 12 w	Experiment 48 w
Experimental group	30	25.33 ± 1.09	27.97 ± 0.96^#^	27.23 ± 1.19^#^
Control group	30	25.17 ± 1.02	25.87 ± 0.94	25.70 ± 0.99
*T*	—	0.587	7.827	5.414
*P*	—	0.559	<0.001	<0.001

*Note.* Comparison with the beginning of the experiment, ^#^*P* < 0.05

**Table 4:** Comparison of ADAS-cog scores before and after intervention between the two groups ($\bar{x}\pm s$).

Group	Number of examples	Start of the experiment	Experiment 12 w	Experiment 48 w
Experimental group	30	16.40 ± 0.93	14.93 ± 1.31^#^	15.00 ± 1.17^#^
Control group	30	16.37 ± 0.93	16.53 ± 0.94	16.90 ± 1.24
*T*	—	0.125	5.435	6.104
*P*	—	0.901	<0.001	<0.001

*Note.* Comparison with the beginning of the experiment, ^#^*P* < 0.05.

## Data Availability

The data used to support the findings of this study are available from the corresponding author upon request.
